# Neural Network-Based Dynamic Segmentation and Weighted Integrated Matching of Cross-Media Piano Performance Audio Recognition and Retrieval Algorithm

**DOI:** 10.1155/2022/9323646

**Published:** 2022-05-13

**Authors:** Tianshu Wang

**Affiliations:** Henan Vocational University of Science and Technology, Zhoukou, Henan 466000, China

## Abstract

This paper presents a dynamic segmentation and weighted comprehensive matching algorithm based on neural networks for cross-media piano performance audio recognition and retrieval. The 3D convolutional neural network process is separated to compress the network parameters and improve the computational speed. Skip connection and layer-wise learning rate solve the problem that the separated network is challenging to train. The piano performance audio recognition is facilitated by shuffle operation. In pattern recognition, music retrieval algorithms are gaining more and more attention due to their ease of implementation and efficiency. However, the problems of imprecise dynamic note segmentation and inconsistent matching templates directly affect the accuracy of the MIR algorithm. We propose a dynamic threshold-based segmentation and weighted comprehensive matching algorithm to solve these problems. The amplitude difference step is dynamically set, and the notes are segmented according to the changing threshold to improve the accuracy of note segmentation. A standard score frequency is used to transform the pitch template to achieve input normalization to enhance the accuracy of matching. Direct matching and DTW matching are fused to improve the adaptability and robustness of the algorithm. Finally, the effectiveness of the method is experimentally demonstrated. This paper implements the data collection and processing, audio recognition, and retrieval algorithm for cross-media piano performance big data through three main modules: the collection, processing, and storage module of cross-media piano performance big data, the building module of audio recognition of cross-media piano performance big data, and the dynamic precision module of cross-media piano performance big data.

## 1. Introduction

In recent years, deep learning has achieved great success in computer vision. 3D convolutional neural networks have been proposed to improve the recognition accuracy based on the recognition of dynamic gestures [1]. The first idea is to train a 3D convolutional neural network using the standard multimodal data training method. Currently, using multimodal data fusion to improve recognition accuracy has become an efficient method; we first train on RGB data, then the generated model is used to fine-tune on depth images and edge images, and finally, the recognition results of multiple modalities are fused; the second one is to use multidirectional feature fusion 3D convolutional neural network, a sequence of images or a short video can be viewed as cubic blocks of video. We use 3D convolution to extract the spatiotemporal features of the image sequence or video from the front, top, and left side, respectively [2]. In this paper, the deep learning method is used in cross-media piano performance audio recognition and retrieval algorithm, making full use of its abstraction ability to learn the correlation between different modal media and proposing a cross-media retrieval method based on a compressed convolutional neural network to improve the retrieval speed based on guaranteeing the retrieval accuracy for the problem of extensive computation and slow pace of deep neural network model.

Traditional cross-media information search is based on the semantic information processing of data in multiple media forms to build a public semantic space and map the data content of various media forms into it. In the public semantic space, supervised classification or unsupervised clustering of cross-media semantic features is performed by machine learning or deep learning algorithms, and feature matching is performed to realize cross-media search. For social networks, it is essential to perform feature mining for cross-media data with unique characteristics purposefully [3]. In addition, bridging the semantic gap between media is necessary to achieve cross-media social network content search under the unique data characteristics of social network multimedia content. On eliminating the semantic sparsity of cross-media social network content, it is essential to effectively use the topic content that reflects the semantic meaning expressed by users and match it with the target topic content to realize cross-media social network content search [4]. Sparse semantic mining and matching of related cross-media information content based on the target topic content information of the query content is the main feature that distinguishes cross-media social network content search from traditional cross-media search. Implementing cross-media social network content search with sparse semantics for target topic content is a domain conventional cross-media extension information search. Practical deep learning algorithms' mining and searching of cross-media content information related to social network security topics have essential theoretical and practical significance for researchers oriented to data mining and information search and regulators, operators, and users in the current social environment. Piano music retrieval refers to the analysis of the content of piano audio to achieve the classification of music archiving and recovery. The extraction of audio features is the basis for the retrieval. In this paper, the system improves the extraction method of various components in the music signal to realize the evaluation of visual playing ability. It achieves the extraction of rhythm, main melody notes, and musical performance of audio.

Given the existing piano performance audio recognition and retrieval algorithms with many attributes, category subdivision, and difficulty in complete coverage and precise refinement, we use artificial intelligence deep learning technology and comprehensive association of piano performance data with multi-dimensional characteristic information and multiple category attribute information to study the extraction and expression of cross-media semantic features of piano performance entities based on deep learning and use piano performance-related data sites and networks as the research objects [5]. Based on the above two research points, we study the cross-media semantic association analysis and extraction of piano performance entities based on the existing multimodal technology data repository and the latest generative adversarial network theory and technology [6]. Combined with the above research content, realize the cross-media audio recognition and retrieval algorithm system based on deep learning, design corresponding experiments to complete the comparison and analysis of the algorithm model indexes of this paper, and conduct the testing of the functional modules designed in this paper.

Since each essential play in piano performance can be regarded as a note event occurrence, note event detection is mainly responsible for detecting note event occurrence, including two subtasks: note start detection and note end detection. By extracting the start time and end time of each note event and considering each note event as a note event segment between the start and end time, complete piano music in WAV format is divided into multiple note event segments, each of which contains one or more notes played at the exact moment. Considering that the onset of some low-frequency messages is usually soft and it is difficult to detect the weak start after the intense onset by traditional methods, this paper proposes to use a combination of band segmentation weighting and power scaling and apply it to spectral flux, which not only enhances the weaker onset and suppresses the more robust onset in the music signal, but also enhances the robustness of the detection method; furthermore, by adding a window differencing process to increase the correctly detected. The overall detection performance is improved by increasing the correct detection of note onsets and reducing false detections through windowing.

## 2. Related Works

Existing cross-media retrieval approaches mainly model different media data to map them into a subspace and then perform similarity measures based on the representations of other media data in the same space [7]. In past research, many approaches used the above ideas to solve cross-media retrieval problems. They can be broadly classified into three categories: subspace-based methods, hash-based methods, and deep learning-based methods [8]. Subspace approaches can learn mapping matrices using pairs of multimedia data information to project different types of media data into a common subspace. Once the multimedia data have a uniform representation, the similarity between the data can be measured directly by calculating the cosine distance or Euclidean distance between the data representations [9]. One of the usual methods is canonical correlation analysis (CCA). For example, Mei et al. proposed clustered canonical correlation analysis to distinguish low-dimensional pictures while maximizing the correlation between two sets [10]. Ren et al. introduced the idea of kernel function into the traditional CCA method [11]. The proposed kernel canonical correlation analysis enhances the ability of CCA to learn nonlinear cross-media correlations. Dhillon et al. offered a typical correlation analysis of multi-label-based, ecclesiastical, and multi-label-based [12]. In addition to the above methods, many other representative methods have been proposed. For example, the advanced semantic association is modeled by a Markov random field-based topic model; the optimal latent space for multimedia data sharing is obtained by joint co-learning latent space and regression methods based on orthogonal constraints, and multimodal data are projected into the latent space [13]. However, whether it is CCA or its extension methods, these methods only maximize the correlation between different media data and do not close the distance between data in the common subspace. The data mapping will produce a particular bias.

Audio codec compression technology is mainly developed by ISO and IEC MPEG organizations. MPEG1 is the first high-quality audio data compression. MPEG1 can be used for up to two audio channels. It features optimal decomposition of the audio signal, adaptive quantization, and entropy coding of adaptive time-frequency blocks (ATFT). Most of the proposed solutions for audio copy detection are based on content fingerprinting [14]. Audio, image, and video fingerprinting has recently become a popular research topic due to the tremendous industry interest in copy detection. Audio fingerprinting refers to compact signatures (extracted from the audio signal) that can distinguish different songs based on their musical content [15]. Traditionally, the proposed audio fingerprinting methods have focused on developing algorithms robust to attacks (effects) such as noise, compression, equalization, and echoes. However, due to the availability of powerful audio editing software, replication detection has become a more complex task that goes far beyond these attacks. Some emerging attacks make pitch shifts and tempo changes. Current research on practical audio algorithms is robust to all content modifications achieved, including noise, compression effects, pitch changes, and tempo changes. In addition, to handle songs and other needs involving short audio segments, audio fingerprinting algorithms are based on the audio signal's local features (fingerprints). A local part represents the audio signal (regardless of the rest of the movement). Many studies on local feature extraction for images and videos have been reported in the literature and have produced powerful and practical algorithms.

With the progress in the field of computer vision research, content-based retrieval techniques have emerged. Yao et al. proposed the combination of scale-invariant feature transform (SIFT) extraction of underlying features and hash retrieval to achieve fast image matching and improve the efficiency of image retrieval [16]. Li et al. combined the grayscale matching algorithm and sifted feature matching algorithm to achieve fast and accurate image matching [17]. The improved method SIFT improves the speed of the algorithm while ensuring the matching accuracy and is also widely used in image retrieval; Baek extracts the content features of music signals and combines them with the semantic description of music to reduce the manual annotation of music retrieval, and improves the retrieval when the hit rate is enhanced [18]. Similarly, in the field of natural language retrieval, with the development of computers and the explosion of information, text retrieval technology has also developed because the text is the closest to semantics. Wu and Ding applied natural language processing technology to text retrieval to extract text semantic features, fully exploit document topic features, and significantly improve the matching with topic tags [19]. However, single-media retrieval still focuses on the underlying components and cannot solve the correlation matching problem between heterogeneous multimedia data to obtain satisfactory cross-media retrieval performance. In addition to single-media retrieval, a combined query method is also proposed. Different media types are mixed for retrieval, and the retrieval result is the same media combination type, which involves multiple modal media. However, it still does not cross the heterogeneous gap of different modal media in essence. The challenge from the press “heterogeneous divide” is drawing more and more attention and has become a hot spot for scholars' research in recent years.

## 3. Neural Network Dynamic Segmentation and Weighted Integrated Matching Model Construction

### 3.1. Neural Network Dynamic Segmentation Model Construction

Fully connected layers implement the traditional neural network structure, and the model is computationally intensive, and the operation is time-consuming. With the introduction of deep learning, deep neural networks have been gradually developed. A deep neural network is a multilayer network structure that divides a target into multiple levels, making the semantic information obtained more sampled and diversified. A convolutional neural network adds a convolutional structure to a deep neural network, which is trained to determine the weights of each connected layer. It then processes the input image to output the category information. The more layers of hidden layers of CNN, the more profound and more complex the network is. Convolutional neural networks have been applied to various fields, and the structure and training algorithm of convolutional neural networks are described below. Convolutional layer: inputting images into a trained CNN will give predicted results. There can be no definite mathematical relationship between the input and output, and its main structure is the convolutional layer. For the input image, the first step is to go through the convolution layer, and the image is viewed as a matrix. The convolution kernel, also called filter, will be preset when doing the convolution operation. The matrix of the same size as the convolution kernel will be selected in turn on the input image to perform the inner product operation with the convolution kernel. The convolution calculation process is shown in Figure 1.

Each convolution kernel extracts only a small portion of the image features, which is also more in line with the way humans process images from a bionic point of view. When humans observe things, they do not need to perceive all aspects, but only the valuable information can be understood, and the elements that are farther away are less relevant. The extracted features are fed into the activation function to obtain the feature map. Different filters are used, and other feature maps are obtained. Usually, after the convolution operation, the size of the output feature map will be smaller than the size of the input image. To make the feature map size more prominent, the input image matrix can be filled with zeros around it, called padding. For an image with matrix size *H* × *W*, a convolution kernel of *E* × *E*, several complementary zeros of *N*, and a convolution step of *S* , the output matrix *H*_1_ × *W*_1_ is

(1) $$\begin{array}{c} H_{1}\times W_{1}=\frac{\sqrt{H-E+2N}}{\sqrt{W-E-2N}}-1. \end{array}$$

Pooling layer: pooling is used to reduce the size of the image. In the extracted feature map, the values between adjacent positions are usually very similar, so the feature map is reduced in dimension without losing too much image information, which prevents the network model from overfitting the training data and reduces the number of parameters of the network model [20]. The input feature map is divided into several small blocks, and the pooling operation is performed on each small image block to shrink the output image by *n* times in each dimension. The everyday pooling operations include average pooling, random pooling, etc. Max Pooling is to select the maximum value of a local image block to represent the local area, just as a school principal can designate a school. Average Pooling is to add all the importance of an image together and take its average to represent the local area, where each value in the local area plays a role. Random pooling is to normalize the values of the input feature map to get the probability value of each deal and then randomly perform the extraction. The larger the probability value, the easier it is to be selected; this pooling method can effectively prevent overfitting. In practical applications, people tend to care more about the most noticeable features in the local area, so the maximum pooling method is used more often. Deep learning methods are used in cross-media piano performance audio recognition and retrieval algorithms, making full use of their abstraction ability to learn correlations between different modal media, and proposing a cross-media retrieval method based on compressed convolutional neural networks to improve retrieval speed on the basis of guaranteed retrieval accuracy in response to the problems of computationally intensive and slow deep neural network models.

(2) $$\begin{array}{c} Z=\frac{\sum \left(w_{1}-x_{1}/b\right)}{f\left(z-1\right)}. \end{array}$$

Connected layer: the fully connected layer is at the end of the convolutional neural network and plays the role of classifying the input. The input image has already been convolved, activated, and pooled, and the fully connected layer integrates all the information for feature classification. In the fully connected layer, the computation process is as follows:

(3) $$\begin{array}{c} a_{1}=\frac{w_{1}\times w_{2}}{2}-\sqrt{w_{3}-b_{1}}. \end{array}$$

Sensation segmentation algorithms based on skin color, contour, motion information, texture, and other information have been studied in-depth and applied to different environmental scenes. Skin color is a feature carried by the human body itself. Skin color-based gesture segmentation becomes the most functional algorithm when the contrast between background and skin color is prominent. In addition, the algorithm has the advantages of simple implementation and high execution efficiency [21]. Before performing gesture segmentation, the skin color model is first established in the color space, and then the skin color ellipse model for static gesture segmentation. However, the main drawback of the skin tone-based gesture segmentation algorithm is that it is less effective when there are near-skin tone targets in the background or when the image contains other skin tone organs such as human faces. Therefore, it is generally mixed with motion information-based and contour-based segmentation algorithms to improve accuracy. Motion information-based gesture segmentation is mainly applied in videos to segment continuously changing dynamic gestures.

The gesture is the primary motion target in the video, and the background is generally stationary. The gesture can be located and segmented from the ground by some motion target detection algorithms. Background subtraction, frame difference, and optical flow methods are the relatively simple and most used motion target detection algorithms. The background subtraction method starts by building a background model. The simplest method is to use the image without the target to be detected as the background and then subtract the pixels of each frame of the video from the background image pixels to find the difference. When the absolute value of the difference is more significant than a predefined threshold, the pixel is determined to belong to the target. Besides, researchers have also proposed some background modeling algorithms, such as the Kalman filtering method, hybrid Gaussian modeling method, and statistical averaging method. The principle of the frame difference method is similar to that of the background subtraction method. The difference is that the frame difference method is to make a difference between adjacent frames in the video. The following equation can express the principle of both. The main challenge of media retrieval is how to solve the problem of data distribution and inconsistency of representation among different media types of data. To this end, the implementation of cross-media retrieval techniques requires the support of multiple technologies, including computer vision, natural language processing techniques, and artificial intelligence.

(4) $$\begin{array}{c} I\left(x,y\right)=\sum_{i=1}x+y/\sqrt{x-y}. \end{array}$$

As a unique feature of human hands, compared with other segmentation methods, gesture segmentation based on contour information can avoid the effects of different racial skin tones and is also robust to illumination changes. The widely used methods are edge detection and contour template matching. The edge detection method obtains the edge of the gesture by the edge detection operator, mainly applicable to images with simple backgrounds. The background edges will enormously interfere with the gesture edges when the environment is more complex. On the other hand, the template matching method locates the gesture by traversing a predefined gesture template over the image to be detected and calculating the match with all the targets on the image. However, due to the variety of gestures, which makes no fixed template for motions, and the high computational cost brought by traversing over the whole image, research scholars gradually give up using the template matching method for gesture segmentation. Gesture segmentation algorithms are also based on active contour models, visual saliency, and entire convolutional neural networks. They have their advantages and disadvantages and are generally a combination of multiple segmentation algorithms to achieve complementary benefits. The advantage of LSTMs over traditional RNNs is that they retain information for more extended periods, allowing for learning earlier information about the sequence, which can significantly impact model decisions. Music is formed by the sequential combination of multiple notes in a time series and the sequence processing properties of LSTMs. This study will apply LSTM networks to learn and train the time series note data and eventually fit music with repetitive melodic structure.

### 3.2. Weighted Integrated Matching Model Construction

The fundamental frequencies obtained by different people humming the same note are different. To make matching under the same criteria, in any case, it is proposed here to use the piano note fundamental frequency as a template, transform the music score into a piano pitch template, and normalize the input music and the piano template by using two templates, the piano template and the input pitch template, which are identical in geometric change trend, for matching, breaking the original graded the idea of matching. The correspondence between standard piano pitches and fundamental frequencies is shown in Table 1. In addition, the bass and treble notes and frequencies in the short score can also be derived from the value of c1.

The problems of start point alignment and note division errors are also avoided. First, the user must hum at least one whole phrase when humming, so a certain length of the template is assumed. Also, the piano templates stored in the database are obtained by dividing the song into whole phrases of variable length. Only full expressions of similar size to the number of notes input are considered, and only the maximum similarity of the entire song is kept. However, when significant errors are encountered in note segmentation, even if the notes that differ between the whole phrase and the input are ignored, it will still result in a minor similarity. The improved DTW algorithm allows the matching of similar profiles and even enables some offset of slices on the time axis. Therefore, the enhanced DTW algorithm is used to solve the errors caused by note segmentation.

## 4. Transmedia Piano Performance Audio Recognition and Retrieval Algorithm Model Design

### 4.1. Cross-Media Piano Performance Audio Recognition Model Design

The audio semantic recognition model is the core of the audio opinion analysis system. The conversion of audio signals to text sequences is achieved by building deep neural network models. Traditional audio recognition systems use Mel-to-spectrum coefficients or linear prediction coefficients as feature vectors, which need to extract acoustic features of single-frequency signals using audio feature extraction algorithms, which are difficult to cover all valid audio information and are susceptible to noise contamination by different signal-to-noise ratios [22]. The audio semantic recognition model proposed in this paper uses the spectrogram of the original speech as input. The features are extracted directly by the convolutional neural network, avoiding the process of multiple conversions of the speech signal in traditional feature extraction methods. The process of generating the spectrogram of the audio signal is shown in Figure 2.

1. Sampling operation is performed on the audio data to obtain the sampled time domain map.
2. The first-order difference of the speech signal increases the amplitude of the high-frequency part to balance the spectrum and alleviate the problem of tilting the range of the speech signal.
3. According to the short-time smooth characteristics of the voice signal to the voice signal for framing processing, set the frame length for 25 ms, the towel shift for 10 ms, the movement in each towel is short-time invariant after split tilt.
4. Use Hamming windows to multiply each frame by a sequence of windows to make the ends of each frame smoother and reduce spectral leakage.
5. The short-time Fourier transform of the speech signal after adding windows to each frame is converted from the time domain to the frequency domain. The modulus is taken as the logarithm to generate the spectrogram.

The first layer of convolution kernel size is 3*∗*3, the number of channels is 32, and the step size is 2. The stride will cause the length of the time and frequency domains to be reduced to half of the input, resulting in a pooling-like effect. The second convolutional layer has a kernel size of 3*∗*3, a channel count of 32, and step sizes of 2 and 1, respectively. The stride will reduce the time-domain length to half of the input while the frequency domain remains unchanged. After the convolutional layer, BatchNorm2d is added to normalize the data to avoid the network instability due to a large amount of data before Hardpan's operation. 2D-CNN extracts the features and inputs the feature representation into the bidirectional GRU network for contextual feature extraction. In this paper, a 7-layer bidirectional GRU is used, and the number of neurons in the hidden layer is set to 1024 to stitch the output of both directions as the output of the GRU. The FC layer fixes the work of the GRU to the 3501-dimensional feature space. Using CTC as the loss function, the gradient of CTC loss is calculated during training, and the model parameters are adjusted by backward transfer to achieve end-to-end training of the whole model. MDCT improved discrete cosine transform is now a commonly used time-frequency transform unit in mainstream audio standard compression and one of the most computationally intensive modules, which has superiority in eliminating boundary noise and improving signal quality, and is a good IMDCT in codec algorithm; it is computationally intensive and calls high-frequency operation steps [23]. Hence, it is suitable for hardware implementation to reduce the processor overhead and power consumption to improve the whole system's performance. This chapter uses DCT-II to propose an efficient algorithm for MDCT and IMDCT for MPEG-1 audio and MPEG-2 international audio coding standards. Finally, the algorithm is compared with the algorithm in this chapter where {*y*(*n*)} is the input data sequence. The following equations give MDCT and IMDCT. For social networks, it is especially important to purposefully feature mine cross-media data with special characteristics. In addition, bridging the semantic gap between media is necessary to achieve cross-media social network content search under the special data characteristics of social network multimedia content.

(5) $$\begin{array}{c} Y=\sum_{n-1}\text{cos}\left(\pi /2n+\sqrt{2k+1}\right), \end{array}$$

where N is the window length and N/2 is the transform coefficient. For simplicity, assume that {*y*(*k*)} is the MDCT coefficient after proper windowing and time-shifting of the original sequence. Usually, it does not correspond to the original data sequence {*y*(*n*)}. An MDCT of length N is typically a power of 2. Assume that N is a multiple of 4. Replacing N-1-n by *n* gives

(6) $$\begin{array}{c} y_{\left(n-1\right)}=\frac{\sqrt{N-n_{1}+1}}{n}. \end{array}$$

The improved MDCT algorithm uses N-1-n to replace the original *n*, forming the following encoding form.

(7) $$\begin{array}{c} Y\left(K\right)=\sum_{n=1}^{n+1}\cos\pi /n\left(2n-2/N\right). \end{array}$$

### 4.2. Analysis of Cross-Media Retrieval Algorithms

In this era of information explosion, human beings are confronted with a massive amount of data and information every day. The traditional single-media search can no longer meet the needs of people's daily operations. Through cross-media retrieval technology, users only need to submit one media type data to get multiple media data related to its content semantics. However, the heterogeneous gap between different media data poses a significant challenge to implementing cross-media retrieval tasks. The solution idea of existing methods is shown in Figure 3. First, the model performs feature extraction for different media data separately. Then, the model maps the projections of different media samples into a unified subspace and thus obtains a suitable representation. Then, the model can use standard distance metrics to calculate and get the similarity between different media samples and achieve cross-media retrieval. In view of the existing piano performance audio recognition and retrieval algorithms, there are many problems, such as wide attribute range, category subdivision, difficult to fully cover, and accurate refinement. Using the deep learning technology of artificial intelligence can comprehensively associate the multidimensional characteristics and multiple category attribute information of piano performance data.

In the above process, the feature extraction and projection mapping of data are particularly critical. Media data has rich semantic information inside, and whether the model can effectively extract the data features will directly affect the final retrieval accuracy. In addition, the model also needs to perform cross-media association learning to complete the projection mapping process accurately [24]. The study of cross-media retrieval methods can promote the development and application of multimedia content understanding theory and meet the demand for cross-media retrieval technology, which has high research application value. At present, the main challenge of cross-media retrieval is how to solve the problem of data distribution and inconsistent representation among different media types of data.

For this reason, the implementation of cross-media retrieval technology requires the support of various technologies, including computer vision, natural language processing techniques, and artificial intelligence. The remainder of this chapter describes the technical principles and knowledge related to cross-media retrieval [25]. Cross-media retrieval involves two different modalities of data, image, and text. The preprocessing of the data has a significant impact on the accuracy of the final cross-media retrieval. For image data, the preprocessing is relatively simple, using an RGB three-layer channel for representation and ensuring the image's uniform size. For text data, its term cannot be used by computer directly, and it can be processed by computer only by converting text data into digital vector form.

## 5. Analysis of Results

### 5.1. Neural Network Dynamic Segmentation and Weighted Integrated Matching Model Analysis

Convolutional neural networks can be divided into two-dimensional convolutional neural networks (2D-CNN) and three-dimensional convolutional neural networks (3D CNN), depending on the convolution method. Different frames of gesture sequence images can be used as other input channels, and then 2D convolutional neural networks are applied. However, 2D convolutional neural networks lack the utilization of inter-frame motion information [26]. In contrast, 3D convolutional neural network methods can compensate for this drawback by entirely using the spatiotemporal feature information between image sequences. In contrast, the structure of 3D convolutional neural networks is more compact. Deep convolutional neural networks are driven by large samples, while the VIVA dataset has only 885 pieces, and fewer samples can lead to overfitting the network during training. Overfitting is manifested by the web having a high recognition rate and low Loss value in the training set but a low recognition rate and high Loss value in the test set. One of the easiest ways to combat overfitting is to augment the samples. The most dominant way of augmentation in the image recognition task is to crop and mirror flip the image spatially. According to the image augmentation, we propose the sample augmentation by time-domain cropping and mirror flip of video data. The comparison of the accuracy of uniformly sampled frames is shown in Figure 4.

This paper is oriented to Hololens for dynamic gesture recognition. Due to the short release time of Hololens glasses, there is limited research related to them, and there is no available public gesture database, so a gesture dataset is constructed called the AMI gesture dataset [27]. From the perspective of ease of use, five quick dynamic gestures were designed: up, down, right, left, and open. The RGB sensor of Hololens was used to capture the five gesture images data, and the sequence images of these five gestures, after grayscale transformation, are shown in Figure 5. To enhance the actual effect of the model, the image data obtained have different backgrounds. Due to the availability of powerful audio editing software, copy detection has become a more complex task that goes far beyond these attacks. Some emerging attacks make pitch shifts and tempo changes. Current research on practical audio algorithms is also robust to all content modifications, including noise, compression effects, pitch changes, and tempo changes. Therefore, complex and straightforward environments were used in the acquisition process to improve the model's accuracy in future practical use. A total of 110K training samples and 10K test samples were finally included, including eight consecutive image frames. The number of negative examples in the training samples was about 95K, and the remaining five gestures were about 3K each. It can be seen that the number of positive and negative examples in the samples is different, but this is also in line with the actual situation because the negative examples are often much more than the positive cases. Still, this sample imbalance is not conducive to network training, so this paper uses resampling techniques in the training process; each of the five gesture samples will be expanded by about 30 times. The number of samples between each piece is approximately equal.

The performance of Kafka and whether it can be used as consistent message architecture can be measured from the perspectives of the ability to transfer data in real-time, whether the file storage mechanism is efficiently implemented, and the effectiveness of practical applications. To improve the efficiency of message lookup in the segment file, improving the current message retrieval algorithm and to implement it can lookup messages more quickly and enhance the Kafka system performance. Since the binary lookup always divides the element from one part into two parts [28]. The time complexity of this search is (log N), which is smaller than the linear O(n). This idea is relatively concise but not efficient for specific scenarios. Based on the concept of a dichotomous lookup algorithm, combined with the elimination and finding of sequences based on the distance difference from the sought value. The system is optimized using a modified dichotomous lookup, which is used to locate the segment in the partition and find the message's logical id in the index file.

### 5.2. Cross-Media Piano Performance Audio Recognition and Retrieval Algorithm Implementation

For audio recognition experiments, the model in this paper uses 128-dimensional log-Mel spectrograms as input features. The 1024-point Short Time Fourier Transform (STFT) is used to extract the spectrograms. It is found that a 7-second-long discourse contains enough emotional information, so if the address is longer than 7 seconds, only the middle part of the length of 7 seconds is calculated. This implementation uses Tensorflow to build the model, using Adam optimizer, with a learning rate of 0.0003 and batch size of 64. The dataset is randomly divided into ten groups, keeping the sentiment distribution constant, eight groups for training, 1 group for validation, and 1 group for testing (fixed test set). The common semantic representation between different modal data is implemented using an adversarial generative network model to achieve cross-media retrieval of scientific and technical resources by spanning the semantic divide between multimodal data. Image and text semantic sharing networks are structurally multilayer, fully connected structures. The front-layer design allows flexible setting of the number of nodes per layer of neurons according to the features of different modalities [29]. Only the fully connected neurons in the last layer are unified to achieve a unified semantic representation of data from different modalities. The training process models learn against each other to optimize the parameters. The convergence of the loss function of the training process is verified. Experiments are conducted on the science and technology resource dataset to obtain the loss curves of the models, and the training process image loss, text loss, and cross-loss are plotted for visualization results. The obtained results are shown in Figure 6, respectively.

It can be seen that in the early training period, the recall accuracy rises faster. With the increase in the number of iterations, the rate of growth in accuracy gradually decreases and finally tends to a steady trend. In the early stage of training, the model's parameters are randomly initialized and cannot fit the data distribution. With the iterations of the training process, the model parameters gradually include the data distribution. In the S&T resource dataset, we can see from the trend of loss distribution that the image feature model converges relatively fast because we use the model parameters pretrained on the large-scale image dataset. To improve the accuracy of segmentation, it is generally mixed with motion information-based and contour-based segmentation algorithms. Motion information-based gesture segmentation is mainly applied in video to do segmentation of continuously changing dynamic gestures. The gradient is continuous because the 12-parameter and cross-entropy are used as the loss function, so the model is fast. The text feature model and the cross-loss feature model also converge gradually with increasing training times. The recall rate of top5 on the training set also increased, and the growth trend slowly leveled off until more than ninety percent. To illustrate the advantages of the proposed algorithm in this paper, the mapped metric is used to measure the performance of different search methods, and the map values are calculated by the top5 and top20 search results of two tasks, text search image, and image search text, on our S&T dataset and this analysis of homo-modal and cross-modal result metrics is compared with CCA, Deep-SM, and CMDN methods. The performance comparison of the experimental results is shown in Figure 7.

The experimental results are the average of nine cross-validations. This experiment uses three metrics, unweighted accuracy (UA), weighted accuracy (WA), and F1 score, to evaluate the model's performance. The experiments are first conducted on the IEMOCAP English dataset using different numbers of inverted residual blocks to verify the recognition effect of other residual blocks. The analysis results show that the model in this paper has a certain degree of improvement in both unweighted accuracy and weighted accuracy compared with the previously commonly used audio emotion recognition models. Compared with the 3D-ACRNN model, the unweighted accuracy of the proposed model is improved by 4.06%; compared with the DNN model, the unweighted accuracy of the proposed model is enhanced by 8.7%; compared with the BCRNN model, the unweighted accuracy of the proposed model is improved by 6.9%. In terms of the number of model parameters, 3D-ACRNN is the model with the most significant number of parameters, with 323.46 M, while the number of parameters of the DNN model is 9.5 M, which is significantly reduced compared with 3D-ACRNN; among the models in the comparison experiments, BCRNN is the model with the smallest number of parameters, with 4.34 M. Compared with the BCRNN model, which has the lowest number of parameters in the reference experiment, the number of parameters is 1.1 M, about one-fourth of the number of parameters of this model. The experiment verifies that the cross-media piano performance audio recognition and retrieval algorithm based on dynamic segmentation and comprehensive weighted matching of neural networks achieves a good recognition effect and effectively reduces the number of parameters of the model. The starting and ending frames of notes can be judged according to the amplitude drop between notes. When the threshold value is fixed, it is determined that the threshold value more significant than the threshold value indicates the start of the message and less than the threshold value indicates the cutoff of the note, which will cause three of the letters to be misjudged as one. The fundamental frequency of the region is averaged to obtain the fundamental frequency when calculating the fundamental frequency. A comparison of the piano performance audio recognition results is shown in Figure 8.

## 6. Conclusion

This paper designs and implements a cross-media piano performance audio recognition and retrieval algorithm based on dynamic segmentation and weighted integrated matching of neural networks. Based on the concept of heterogeneous neural networks, this paper designs the technical solutions of the cross-media piano performance audio recognition system building module, the retrieval algorithm system data processing module, the audio recognition analysis system analysis module, and the retrieval algorithm analysis system module, respectively. Based on the design of the technical system scheme, the critical functional modules of the audio recognition analysis system and the implementation details of the algorithm logic are elaborated. Finally, the system testing process is carried out to verify the usability of the neural network-based audio recognition system. This paper focuses on the problem of matching accuracy in music retrieval algorithms, proposes an algorithm for note segmentation with a dynamic threshold to improve note segmentation accuracy, establishes a similarity matching algorithm with the weighted synthesis of basic piano templates, increases the fault tolerance mechanism of matching, and enhances the robustness and adaptability of the algorithm. This paper conducts a comprehensive analysis, comparison, and optimization of existing message retrieval algorithms. The shortcomings of current retrieval algorithms are found, and an improved message queue retrieval algorithm is designed and implemented to improve the system efficiency. The average number of lookups is significantly better than the existing message retrieval algorithm, and it can complete the message retrieval of Kafka efficiently and accurately. The performance of the improved message retrieval algorithm is also compared in terms of mathematical reasoning and the number of lookups, and the enhanced message retrieval algorithm is proved to be effective and efficient in practice.

## Figures and Tables

**Figure 1:** Convolutional neural network operation process.

**Figure 2:** Network structure of audio recognition model.

**Figure 3:** Cross-media retrieval implementation process.

**Figure 4:** Comparison of the accuracy of uniformly sampled frames.

**Figure 5:** Transformed data set.

**Figure 6:** Loss plot of the variation of the loss function.

**Figure 7:** Experimental results performance comparison.

**Figure 8:** Comparison of piano performance audio recognition results.

**Table 1:** Correspondence table of scale and frequency.

Scale	c1	d1	e1	f1	g1	a1	b1

Simple score	1	2	3	4	5	6	7

Frequency (Hz)	267	281	319	354	398	423	453

Scale	c1	d1	e1	f1	g1	a1	b1

Simple score	1	2	3	4	5	6	7

Frequency (Hz)	324	341	431	445	487	465	532

Scale	c1	d1	e1	f1	g1	a1	b1

Simple score	1	2	3	4	5	6	7

Frequency (Hz)	375	398	425	478	496	497	564

## Data Availability

The data used to support the findings of this study are available from the corresponding author upon request.
